The article "Fluoride exposure and intelligence in school-age children: evidence from different windows of exposure susceptibility" was retracted in 2022. Reasons: errors in the analysis; errors in the results or conclusions; concerns about the data.

# Fluoride exposure and intelligence in school-age children: evidence from different windows of exposure susceptibility

**DOI:** 10.1186/s12889-020-09765-4

**Published:** 2020-11-04

**Authors:** Kaihong Xu, Ning An, Hui Huang, Leizhen Duan, Jun Ma, Jizhe Ding, Tongkun He, Jingyuan Zhu, Zhiyuan Li, Xuemin Cheng, Guoyu Zhou, Yue Ba

**Affiliations:** 1 Department of Environmental Health, School of Public Health, Zhengzhou University, Zhengzhou, 450001 Henan China; 2 Environment and Health Innovation Team, School of Public Health, Zhengzhou University, Zhengzhou, 450001 Henan China; 3 Department of Medical Services, Zhengzhou Central Hospital Affiliated to Zhengzhou University, Zhengzhou, 450001 Henan China; 4 Department of Endemic Disease, Kaifeng Center for Disease Control and Prevention, Kaifeng, 475000 Henan China; 5 The Medical Section, The Eighth People Hospital of Zhengzhou, Zhengzhou, 450000 Henan China; 6 Yellow River Institute for Ecological Protection & Regional Coordinated Development, Zhengzhou University, Zhengzhou, 450001 Henan China

**Keywords:** Fluoride, Prenatal, Childhood, Intelligence

## Abstract

**Background:**

The intellectual loss induced by fluoride exposure has been extensively studied, but the association between fluoride exposure in different susceptibility windows and children’s intelligence is rarely reported. Hence, we conducted a cross-sectional study to explore the association between fluoride exposure in prenatal and childhood periods and intelligence quotient (IQ).

**Methods:**

We recruited 633 local children aged 7–13 years old randomly from four primary schools in Kaifeng, China in 2017. The children were divided into four groups, of which included: control group (CG, *n* = 228), only prenatal excessive fluoride exposure group (PFG, *n* = 107), only childhood excessive fluoride exposure group (CFG, *n* = 157), both prenatal and childhood excessive fluoride exposure group (BFG, *n* = 141). The concentrations of urinary fluoride (UF) and urinary creatinine (UCr) were determined by fluoride ion-selective electrode assay and a creatinine assay kit (picric acid method), respectively. The concentration of UCr-adjusted urinary fluoride (CUF) was calculated. IQ score was assessed using the second revision of the Combined Raven’s Test-The Rural in China (CRT-RC2). Threshold and saturation effects analysis, multiple linear regression analysis and logistic regression analysis were conducted to analyze the association between fluoride exposure and IQ.

**Results:**

The mean IQ score in PFG was respectively lower than those in CG, CFG and BFG (*P* < 0.05). The odds of developing excellent intelligence among children in PFG decreased by 51.1% compared with children in CG (*OR* = 0.489, 95% *CI*: 0.279, 0.858). For all the children, CUF concentration of ≥1.7 mg/L was negatively associated with IQ scores (*β* = − 4.965, 95% *CI*: − 9.198, − 0.732, *P* = 0.022). In children without prenatal fluoride exposure, every 1.0 mg/L increment in the CUF concentration of ≥2.1 mg/L was related to a reduction of 11.4 points in children’s IQ scores (95% *CI*: − 19.2, − 3.5, *P* = 0.005).

The article "Fluoride exposure and intelligence in school-age children: evidence from different windows of exposure susceptibility" was retracted in 2022. Reasons: errors in the analysis; errors in the results or conclusions; concerns about the data.

**Conclusions:**

Prenatal and childhood excessive fluoride exposures may impair the intelligence development of school children. Furthermore, children with prenatal fluoride exposure had lower IQ scores than children who were not prenatally exposed; therefore the reduction of IQ scores at higher levels of fluoride exposure in childhood does not become that evident.

## Background

Fluoride can prevent dental caries [1], and it is beneficial to bone metabolism as an essential trace element in the body [2]. However, the safe dose range of fluoride is limited [3]. Increasing evidences have shown that long-term exposure to excessive fluoride will not only increase the risk of dental fluorosis [4] and skeletal fluorosis [5], but also impair neural development by influencing gene and protein expression, enzyme activity and inducing oxidative stress [6].

The effects of fluoride on the nervous system have been manifested in intellectual development of rats [7]. Chronic high fluoride exposure of maternal mice in drinking water during pregnancy and lactation may have harmful influences on learning and memory of young mice [8]. Studies indicated that fluoride ingested by the mother can cross the placental barrier [9] and the blood-brain barrier [10], to affect the offspring’s cognitive function development [11]. Green et al. (2019) found that prenatal exposure to excessive fluoride was associated with children’s lower IQ scores. Surprisingly, the mean fluoride concentrations of drinking water in the fluoridated and non-fluoridated communities were 0.59 and 0.13 mg/L, respectively [12], which were lower than 1.5 mg/L suggested by the World Health Organization [3]. Elsewhere, a cross-sectional study in India showed that children’s intelligence quotient (IQ) was inversely associated with fluoride exposure via drinking water and maternal diet during pregnancy [13]. And, another Mexican study suggested that maternal exposure to excessive fluoride during pregnancy reduced children’s cognition and IQ scores, and the fluoride exposure range was 0.15–1.38 mg/L [14]. Some contradictory results have been found in the association between childhood fluoride exposure and intellectual development. Among such instances, a Chinese study found that exposure to moderately high fluoride in childhood could cause the loss of excellent intelligence [15]. A cohort study in Canada also reported that water fluoride concentration was associated with intelligence loss of formula-fed children, and the mean fluoride concentrations in the drinking water in the fluoridated and non-fluoridated communities appeared same as the study of Green et al. (2019) [16]. Meanwhile, no association between excessive fluoride and IQ scores were observed in a community water fluoridation program in New Zealand, where the fluoride concentration ranged from 0.7 to 1.0 mg/L [17]. Adding to the above, there was no significant correlation between fluoride exposure and lower IQ in adolescents [18]. Due to the different study populations and areas, the conclusion that excessive fluoride causes loss of children’s IQ still lacks strong evidence. Furthermore, compared with children without tobacco smoke exposure history, the relative risk of behavior problems of children exposed only in prenatal period was 90% higher, while that of children exposed only in postnatal period was 30% according to a prospective birth cohort study [19], indicating that the effects of prenatal and postnatal exposure on children’s neurodevelopment are different.

The article "Fluoride exposure and intelligence in school-age children: evidence from different windows of exposure susceptibility" was retracted in 2022. Reasons: errors in the analysis; errors in the results or conclusions; concerns about the data.

On the basis of the above analyses, it is an urgent need to distinguish the health effects of fluoride exposure in different susceptibility windows during development. Here, we selected Tongxu County, Kaifeng, Henan Province, a typical drinking-water-born fluorosis area, as the research region (no industrial sources of neurotoxic environmental pollutants such as arsenic, lead, mercury, etc.) to assess the association between excessive fluoride exposure in prenatal or childhood periods and children’s intelligence.

## Methods

### Study areas and population

Four primary schools were randomly selected in Tongxu County, Henan Province, China from late April to late May in 2017. The study was conducted in the middle of the semester, when students were in school with no psychological fluctuations caused by the beginning or end of the semester and psychological pressure brought by the final exam. The natural conditions, living conditions, population composition, living habits and dietary structure of the four schools were consistent, and no industrial fluoride pollution source was found in all the investigated areas. Exclusion criteria included taking calcium supplements, children who were not resident locally, diagnosed of digestive disease, thyroid disease, calcium and phosphorus metabolism disorders. The potential eligible participants included 642 students (7–13 years old) from the four primary schools in grades 2–6, and were recruited by the cluster sampling method. Then, 9 children were excluded for incomplete information or urinary samples. Finally, a total of 633 participants were included in the study with the participation rate of 98.60%. This study was approved by the Ethics Review Board at Zhengzhou University (ZZUIRB2017–018). All the children and their legal guardians were informed of the study procedures and signed the informed consent before recruitment.

The article "Fluoride exposure and intelligence in school-age children: evidence from different windows of exposure susceptibility" was retracted in 2022. Reasons: errors in the analysis; errors in the results or conclusions; concerns about the data.

### General data collection

The study’s questionnaire was designed in advance, including sociodemographic information, medical history, maternal pregnancy and delivery information, birth characteristics and personal behaviors (such as daily exercise, diet). The student’s status at school was filled by the student or the teacher, and other information was provided by the guardian. The physical measurements of this study were completed by the clinical professional doctors in the survey area based on the standard method recommended by Chinese hygiene department. Physical measurements included weight, height, etc. The height and weight of the participants were measured by standard calibrated ruler and weight measurement device (V. BODY HBF-371; OMRON, Kyoto, Japan) according to the operation guidance, and were measured twice to the nearest 0.1 cm and 0.1 kg, respectively, all done while the participants wore light clothing and stood barefooted. The average value was considered for analysis. Body mass index (BMI) was calculated according to weight (kg)/square of height (m^2^).

### Exposure assessment

Morning urine (at least 50 mL) was collected into cleaned polyethylene tubes and then stored at − 80 °C, as described in the previous study [20]. Determination of urinary fluoride (UF) concentrations were conducted by a fluoride ion-selective electrode (Shanghai Exactitude Instruments, Shanghai, China), and the standard curve method was used according to the protocol of health industry standard of China (WS/T 89–2015). The fluoride standard stock solution (National Center for Analysis and Testing for Nonferrous Metals and Electronic Materials, GSB 04–1771-2004) was 1000 mg/L. UF levels in each sample were measured twice, and the mean value was used. The recovery rates reached 93.19–109.93%. The concentrations of urinary creatinine (UCr) were determined using a creatinine assay kit (picric acid method) (Jiancheng Bioengineering Institute, Nanjing, China). All of the samples were measured in duplicate, and two measurements were averaged for analysis. Fifteen percent of urine samples from different plates were randomly selected to repeat the measurement of UCr. The recovery rates were 93.83–105.25%. To correct the influence of urinary dilution on UF concentration, the concentrations of UCr-adjusted urinary fluoride (CUF) were calculated using the following equation: CUF (mg/L) = (UF (mg/L)/UCr (mg/L)) × UCr_mean_ (mg/L), where UCr_mean_ is the mean Cr concentration of total samples available [21]. According to whether the mother was exposed to excessive fluoride (the fluoride concentration in drinking water > 1.0 mg/L, GB5749–2006) during pregnancy, the children were divided into two groups: prenatal excessive fluoride exposure group (PF), and prenatal control group (PC). Moreover, according to whether the children’s UF concentration exceeded the national standard (UF concentration > 1.4 mg/L, WS/T 256–2005), children were divided into childhood excessive fluoride exposure group and childhood control group. On the basis of the above criteria, eligible children were divided into four groups: only prenatal excessive fluoride exposure group (PFG), only childhood excessive fluoride exposure group (CFG), both prenatal and childhood excessive fluoride exposure group (BFG), control group (CG).

The article "Fluoride exposure and intelligence in school-age children: evidence from different windows of exposure susceptibility" was retracted in 2022. Reasons: errors in the analysis; errors in the results or conclusions; concerns about the data.

### Outcome assessment

The second revision of the Combined Raven’s Test-The Rural in China (CRT-RC2) was used to measure children’s IQ scores [22]. The IQ test was conducted in the school classrooms. Each child had an independent desk. Students completed the answer sheets independently under the supervision of trained investigators. The test conditions, test methods, calculation steps, etc. performed were totally consistent with the protocol of the Combined Raven's Test. The classification criteria for children’s IQ were excellent (IQ scores ≥130), superior (IQ scores 120–129), high normal (IQ scores 110–119), normal (IQ scores 90–109), dull normal (IQ scores 80–89), marginal (IQ scores 70–79) and retarded (IQ scores ≤69) [23]. Due to few children with IQ scores < 90 (*n* = 11), thus, we included children with IQ scores ≥90 (*n* = 622) in the intelligence analysis.

### Statistical analysis

Epidata version 3.0 (Epidata Association Odense, Denmark) was used to establish the database, and all data were independently integrated into the database by two investigators. One-way ANOVA was used to compare the difference of the continuous variables among the four exposure groups and the results were described by the mean ± standard deviation. Chi-square test was used to compare the difference of distribution of categorical variables in different groups, and the results were described in percentage (number). Multiple logistic regression analysis was conducted to explore the differences of intelligence distribution in different fluoride exposure groups. Threshold and saturation effects analysis and multiple linear regression analysis were used to analyze the association between CUF concentration and IQ scores and, the association between prenatal fluoride exposure and IQ scores. The analyses were adjusted for children’s age, gender, gestational weeks, maternal education level, paternal education level and children’s BMI. All data were analyzed by SPSS software, version 25.0 (SPSS Inc., Chicago, USA) and EmpowerStats (R). Plots were drawn by Graphpad prism 6.01. The criterion with statistical difference was *P* < 0.05.

The article "Fluoride exposure and intelligence in school-age children: evidence from different windows of exposure susceptibility" was retracted in 2022. Reasons: errors in the analysis; errors in the results or conclusions; concerns about the data.

## Results

### Distribution of general characteristics

All of the 633 children were divided into CG, PFG, CFG and BFG. As shown in Table 1, children’s age in PFG and BFG were higher than that in CG and CFG (*P* < 0.05, respectively). Similar results could be observed in the distribution of children’s height, weight and BMI (*P* < 0.05, respectively). The CUF concentrations of children in PFG, CFG and BFG were higher than that in CG, and the CUF concentrations of children in CFG and BFG were higher than that in PFG (*P* < 0.05, respectively). IQ scores of children in PFG were lower than that in CG, CFG and BFG (*P* < 0.05, respectively). Moreover, no statistical differences were observed among the four groups under the distribution of children’s gender, birth weight, gestational weeks, maternal and paternal education levels and birth mode (*P* > 0.05, respectively).

**Table 1:** Characteristics of children aged 7–13 years

Variables	CG(*n* = 228)	PFG(*n* = 107)	CFG(*n* = 157)	BFG(*n* = 141)	*F*/*χ*^2^	*P*^f^
Age (years)^d^	9.66 ± 1.29	10.68 ± 1.16^a^	9.76 ± 1.24^b^	10.33 ± 1.25^abc^	21.249	< 0.001
Gender^e^					1.500	0.682
Boys	49.1(112/228)	42.1(45/107)	47.8(75/157)	46.8(66/141)		
Girls	50.9(116/228)	57.9(62/107)	52.2(82/157)	53.2(75/141)		
Height (cm)^d^	138.42 ± 9.81	144.04 ± 9.33^a^	137.56 ± 8.96^b^	142.44 ± 8.96^ac^	15.624	< 0.001
Weight (kg)^d^	33.36 ± 8.69	37.63 ± 8.97^a^	32.27 ± 6.49^b^	36.51 ± 7.85^ac^	13.811	< 0.001
BMI (kg/m^2^)^d^	17.17 ± 2.68	17.99 ± 3.14^a^	16.93 ± 2.36^b^	17.82 ± 2.50^ac^	5.112	0.002
Birth weight (kg)^d^	3.36 ± 0.59	3.35 ± 0.39	3.38 ± 0.53	3.35 ± 0.46	0.090	0.965
CUF (mg/L)^d^	0.82 ± 0.30	0.98 ± 0.29^a^	2.05 ± 0.58^ab^	2.13 ± 0.59^ab^	378.736	< 0.001
IQ scores^d^	123.92 ± 12.50	119.76 ± 11.28^a^	124.65 ± 10.88^b^	123.04 ± 11.24^b^	4.139	0.006
Maternal age of pregnancy (y)^d^	26.72 ± 4.95	25.51 ± 3.80^a^	25.30 ± 3.81^a^	25.70 ± 4.16^a^	3.637	0.013
Gestational weeks (w)^d^	36.98 ± 4.71	36.97 ± 4.95	37.19 ± 3.86	38.01 ± 3.76	1.363	0.253
Paternal education level (y)^e^					2.661	0.850
Primary school or below	9.0(19/210)	7.0(7/100)	6.7(10/149)	9.2(12/131)		
Junior high school	69.0(145/210)	71.0(71/100)	74.5(111/149)	66.4(87/131)		
High school or above	21.9(46/210)	22.0(22/100)	18.8(28/149)	24.4(32/131)		
Maternal education level (y)^e^					8.583	0.198
Primary school or below	18.0(37/206)	10.0(10/100)	12.7(19/150)	10.2(13/128)		
Junior high school	59.7(123/206)	73.0(73/100)	68.7(103/150)	68.0(87/128)		
High school or above	22.3(46/206)	17.0(17/100)	18.7(28/150)	21.9(28/128)		
Birth mode^e^					8.525	0.202
Natural labour	64.5(140/217)	75.7(81/107)	63.5(99/156)	72.9(97/133)		
Cesarean delivery	35.0(76/217)	24.3(26/107)	35.3(55/156)	26.3(35/133)		
Rest	0.5(1/217)		1.3(2/156)	0.8(1/133)		

^a^*P* < 0.05 compared to CG

^b^*P* < 0.05 compared to PFG

^c^*P* < 0.05 compared to CFG

^d^Data was presented as the mean ± standard deviation for continuous variables

^e^Data was presented as the percentage (number) for categorical variables

^f^Variance analysis was used to compare the differences of continuous variables, and Chi-square test was performed to compare the differences of categorical variables

The article "Fluoride exposure and intelligence in school-age children: evidence from different windows of exposure susceptibility" was retracted in 2022. Reasons: errors in the analysis; errors in the results or conclusions; concerns about the data.

### Comparisons of intelligence in different fluoride exposure groups

Logistic regression analysis suggested that the odds of developing excellent intelligence for children in PFG decreased by 51.1% compared with children in CG (*OR* = 0.489, 95% *CI*: 0.279, 0.858). No significant associations between the odds of developing normal, high normal and superior intelligence and fluoride exposure were found (Table 2). As shown in Fig. 1, the percentages of children with superior intelligence in PFG and BFG were 34 and 35%, respectively. Children with excellent intelligence in CG and CFG had the percentage of 33 and 34%, respectively.

**Table 2:** Logistic regression analysis between fluoride exposure and children’s intelligence

	Normal		High normal		Superior		Excellent	
	*OR* (95%*CI*)	*P*	*OR* (95%*CI*)	*P*	*OR* (95%*CI*)	*P*	*OR* (95%*CI*)	*P*
CG (*n* = 223)	reference		reference		reference		reference	
PFG (*n* = 104)	1.334(0.716,2.486)	0.364	1.478(0.869,2.514)	0.149	1.109(0.676,1.820)	0.683	0.489(0.279,0.858)	0.013
CFG (*n* = 155)	0.593(0.305,1.152)	0.123	1.226(0.756,1.987)	0.409	1.041(0.670,1.616)	0.858	1.037(0.671,1.603)	0.869
BFG (*n* = 140)	0.881(0.473,1.638)	0.688	1.262(0.769,2.072)	0.357	1.177(0.752,1.842)	0.476	0.738(0.462,1.179)	0.204

**Fig. 1:** Distribution of all children’s intelligence in different fluoride exposure groups. The percentages of children with superior intelligence in PFG and BFG were 34 and 35%, respectively. Children with excellent intelligence in CG and CFG had the percentage of 33 and 34%, respectively

### Association between CUF concentration and children’s IQ scores

The CUF concentrations of the 633 children included in the study ranged from 0.18 mg/L to 3.39 mg/L, and the mean ± standard deviation was 1.44 ± 0.76 mg/L. The range of IQ scores was 60.00–146.00, and the mean ± standard deviation was 122.48 ± 12.91. In Fig. 2, we observed a negative association between children’s IQ scores and concentrations of CUF at ≥1.7 mg/L (*P* < 0.05).

The article "Fluoride exposure and intelligence in school-age children: evidence from different windows of exposure susceptibility" was retracted in 2022. Reasons: errors in the analysis; errors in the results or conclusions; concerns about the data.

**Fig. 2:** Association between fluoride exposure and children’s IQ scores of all children^a^. ^a^ Adjusted for age, gender, gestational weeks, maternal education level, paternal education level and children’s BMI. The estimated values and their corresponding 95% *CI* were respectively represented by the solid line and the dotted lines. A negative association was observed between children’s IQ scores and concentrations of CUF at ≥ 1.7 mg/L (*P* < 0.05)

Multiple liner regression analysis presented that a decrease of 4.965 points in children’s IQ scores was associated with each 1.0 mg/L increase in the CUF concentration of ≥1.7 mg/L (95% *CI*: − 9.198, − 0.732, *P* = 0.022) (Table 3). No statistical significance was observed in the association between CUF concentration and children’s IQ scores in PF and PC, respectively. Furthermore, the interaction between prenatal exposure and CUF concentration on children’s IQ scores in PF and PC was not statistically significant (*P* > 0.05, respectively) (Table 3).

**Table 3:** Multiple liner regression analysis between fluoride exposure and children’s IQ scores

	< 1.7 mg/L			≥ 1.7 mg/L		
	*n*	*β* (95% *CI*)	*P*	*n*	*β* (95% *CI*)	*P*
Total^a^	430	2.785(−0.832,6.403)	0.131	203	−4.965(−9.198, −0.732)	0.022
PF^a^	148	4.054(−3.169,11.277)	0.268	100	−3.929(−9.396,1.538)	0.156
PC^a^	282	3.146(−1.138,7.430)	0.149	103	−6.595(−13.323,0.133)	0.055
*P* for Interaction^b^			0.651			0.726

^a^Adjusted for age, gender, gestational weeks, maternal education level, paternal education level, children’s BMI

^b^Adjusted for age, gender, gestational weeks, maternal education level, paternal education level, children’s BMI, group (PF or PC), CUF

### Threshold and saturation effects of fluoride exposure on children’s IQ scores in PF and PC

Figure 3a showed that the association between CUF concentrations and changes in IQ scores among children in PF was initially positive, and then saturated gradually. However, in Fig. 3b, children’s IQ scores in PC rose slowly to a peak and then fell evidently. And we observed every 1.0 mg/L increment in the CUF concentration of ≥2.1 mg/L was related to a reduction of 11.4 points in children’s IQ scores (*β* = − 11.4, 95% *CI*: − 19.2, − 3.5, *P* = 0.005) (Fig. 3b).

**Fig. 3:** Associations between fluoride exposure and children’s IQ scores in PF (**a**)^a^ and PC (**b**)^a^. ^a^ Adjusted for age, gender, gestational weeks, maternal education level, paternal education level and children’s BMI. The estimated values and their corresponding 95% *CI* were represented by the solid line and the dotted lines

The article "Fluoride exposure and intelligence in school-age children: evidence from different windows of exposure susceptibility" was retracted in 2022. Reasons: errors in the analysis; errors in the results or conclusions; concerns about the data.

## Discussion

Our study examined the association between excessive fluoride exposure in prenatal and childhood periods and the intelligence of school-age children. We found that prenatal excessive fluoride exposure could cause lower IQ scores, especially the decreased odds of developing excellent intelligence. Meanwhile, a negative association between fluoride exposure and children’s IQ scores was observed in children without prenatal exposure.

Several epidemiological studies have shown that excessive prenatal fluoride exposure could reduce offspring’s IQ scores [12, 14], which are consistent with our findings. Fluoride ingested by the mother during pregnancy can cross the placental barrier and enter the embryo [24], and affect the brain development of children [25]. In addition, we found that the odds of developing excellent intelligence for children in PFG decreased by 51.1% compared with nonexposed children. Lower intelligence has become a new public health and social problem, which not only endangers children’s physical and mental health, but also increases family burden [26, 27]. Hence, it is necessary to consider limiting the intake of excessive fluoride by pregnant women.

For all participants, we observed that a decrease of 4.965 points in children’s IQ scores was associated with each 1.0 mg/L increase in the CUF concentration of ≥1.7 mg/L. A cross-sectional study found that moderate fluoride exposure was inversely correlated with children’s IQ scores, and suggested a UF threshold of 1.6 mg/L for intelligence damage [15]. The reason for the difference between the two thresholds may be that we adjusted the UF concentration by UCr. We further found that every 1.0 mg/L increment in the CUF concentration of ≥2.1 mg/L was related to a reduction of 11.4 points of children’s IQ scores in prenatal control group. These results suggested that excessive fluoride exposure in childhood was negatively associated with children’s IQ scores. Fluoride can penetrate into the brain through the blood-brain barrier [10]. Several researches reported that exposure to fluoride could damage the function of hippocampus and thyroid, thus impairing intellectual development of school children [28, 29]. Contrary, no findings were obtained in a New Zealand study to support that fluoride exposure in community water fluoridation could affect neurologic development or IQ of children aged 7–13 years old [17]. Also, a study in India showed that fluorosis was not significantly associated with adolescent intelligence in a non-endemic fluorosis area with lower level of fluoride [18]. The differences of exposure level, ethnicity and study areas may explain these results which are inconsistent with ours.

The article "Fluoride exposure and intelligence in school-age children: evidence from different windows of exposure susceptibility" was retracted in 2022. Reasons: errors in the analysis; errors in the results or conclusions; concerns about the data.

An animal experiment found that fluoride may elevate fluoride tolerance by down-regulating ribosomes, pancreatic secretion, steroid biosynthesis, glutathione metabolism, steroid biosynthesis, and glycerolipid metabolism gene expression [30]. Furthermore, another animal experiment suggested that the decrease of the susceptibility to fluoride was related to the changes in expression level of glutathione S-transferase gene after fluoride stimulation [31]. In the current population study, we found some similar results. Children with prenatal fluoride exposure have lower IQ scores, and therefore the reduction of IQ scores at higher CUF levels in some range during childhood did not become that evident. In addition, the IQ scores of children without prenatal exposure decreased evidently with the increase of CUF concentrations of ≥2.1 mg/L (Fig. 3). However, the mechanism still needs to be further studies at the population level.

Our study has several limitations. Firstly, urine samples were collected in the morning, not 24 h. However, a study has reported that for population studies, morning urine is a good representation of 24-h urine samples and the results are reliable [32]. Secondly, considering the influence of urine dilution on UF, UCr was used to adjust the UF. However, due to the instability of UCr in growing children or experiencing puberty, this may also be one of the limitations. Since the subjects in our study are all boarding students, their same diet and sleep schedule could alleviate the limitation to some extent. Thirdly, it was very difficult to obtain UF concentrations data from a pregnant mother, thus, we used the fluoride level in local drinking water during mother’s pregnancy. This is because fluoride level in drinking water is highly correlated with UF level [33]. On point, all the mothers in the study were local residents, and local drinking water fluoride level in the village could well represent maternal fluoride exposure level. Fourthly, the project was a cross-sectional study which lasted 1 month, and only one-time sampling was conducted, and so the inferential causality was weak. Long term large-scale epidemiological studies should be conducted to provide more abundant evidences. Finally, we tried to reduce the influence on the results through adjusting for children’s age, gender, gestational weeks, parental education levels and children’s BMI, though some unknown confounding factors may still.

The article "Fluoride exposure and intelligence in school-age children: evidence from different windows of exposure susceptibility" was retracted in 2022. Reasons: errors in the analysis; errors in the results or conclusions; concerns about the data.

## Conclusions

In summary, prenatal and childhood exposure to excessive fluoride may impair the intelligence development of school children. Furthermore, children with prenatal fluoride exposure had lower IQ scores than children who were not prenatally exposed; therefore the reduction of IQ scores at higher levels of fluoride exposure in childhood does not become that evident. Our results support the necessary restriction of fluoride intake for pregnant women and school-age children to protect children’s intellectual development.

## Data Availability

The datasets used and/or analyzed during the current study are available from the corresponding author on reasonable request.

## Abbreviations

IQ: Intelligence quotient
BMI: Body mass index
UF: Urinary fluoride
UCr: Urinary creatinine
CUF: UCr-adjusted urinary fluoride
PF: Prenatal excessive fluoride exposure group
PC: Prenatal control group
PFG: Only prenatal excessive fluoride exposure group
CFG: Only childhood excessive fluoride exposure group
BFG: Both prenatal and childhood excessive fluoride exposure group
CG: Control group
CRT-RC2: The second revision of the Combined Raven’s Test-The Rural in China
CI: Confidence interval
